The article "Quantitative Diagnosis of TCM Syndrome Types Based on Adaptive Resonant Neural Network" was published in 2022. Journal: Comput Intell Neurosci.

# Quantitative Diagnosis of TCM Syndrome Types Based on Adaptive Resonant Neural Network

**DOI:** 10.1155/2022/2485089

**Published:** 2022-06-24

**Authors:** Yue Zhao, Yuandi Huang

**Affiliations:** School of Chinese Medicine, Hong Kong Baptist University, Hong Kong 999077, China

## Abstract

Artificial intelligence has become one of the most rapidly developing disciplines in the application field of pattern recognition. In target recognition, sometimes, there are multiple identical or similar copies of the target to be recognized in the image, and it is difficult to classify and estimate by traditional methods. In this case, it is necessary to use the SOM network to separate multiple targets and use the multiple order parameters in the improved SNN to pair the target. The change of its thickness can intuitively reflect the abnormality of its tissue. Therefore, the choroidal thickness of the central fovea can be measured to study the relationship between the choroidal structure and BRVO and arteriosclerosis. The purpose of this study is to further study the correlation between branch retinal vein occlusion and arteriosclerosis by quantitatively measuring retinal vessel diameter and choroidal thickness, to analyze the correlation between different TCM syndrome types of nonischemic BRVO and retinal arteriosclerosis, and to provide theoretical basis for clinical nonischemic BRVO TCM syndrome types and traditional Chinese medicine treatment, so as to reflect its clinical application value. In order to solve the single fixed structure of traditional SNN and poor scalability, combined with the Kohonen layer structure in the self-organizing mapping network, an improved collaborative neural network model is proposed. This paper studies the network training method and operation convergence and analyzes the converged network and the pattern classification results obtained by the network. In order to solve the single fixed structure of traditional SNN and poor scalability, combined with the Kohonen layer structure in the self-organizing mapping network, an improved collaborative neural network model is proposed. The results of our proposed improved model on the MNIST dataset can achieve the same level of current state-of-the-art machine learning classifiers in recognition accuracy with a smaller network size and network complexity.

## 1. Introduction 

In the occurrence of retinal vein occlusion, a large number of studies have confirmed that arteriosclerosis is a high-risk factor for its occurrence [1]. In some studies, homocysteine is found to be an independent factor leading to arteriosclerosis. Homocysteine, or homocysteine, is a sulfur-containing amino acid, which is mainly converted from methionine in the body and is an intermediate product of the methionine cycle. In addition, it can synthesize methionine again with the participation of folic acid [2]. Studies have shown that elevated homocysteine is an independent risk factor for arteriosclerosis, and its mechanisms include homocysteine that can lead to endothelial cell hypertrophy and injury, mainly because homocysteine reduces endothelial-dependent vasodilation responses. Endothelial function is damaged; superoxide anion, hydroxyl radicals, and hydrogen dioxide can be generated during homocysteine oxidation, which can further damage endothelial cells; homocysteine induces oxidative stress by reducing the activity of some enzymes in the body [3]. Homocysteine can also induce the proliferation of smooth muscle cells in the middle of the blood vessels, and by activating related proteases, a series of reactions are generated, and finally the apoptosis of smooth muscle cells is induced [4].

There are a lot of studies on the relationship between homocysteine and branch retinal vein occlusion, but the relationship between homocysteine and branch retinal vein occlusion is controversial, and some studies have proved that homocysteine is an independent risk of branch retinal vein occlusion factor, but other studies have not found this relationship [5–8]. There is a study to investigate the changes in plasma homocysteine levels in patients with branch retinal vein occlusion during acute and convalescent phases [9]. In patients with branch retinal vein occlusion, the plasma homocysteine level gradually increased from the acute phase to the recovery phase after venous occlusion, reached a peak one month after the occurrence of venous occlusion, and then gradually decreased in 6 months after the occurrence of BRVO To normal levels. This change was independent of plasma vitamin B12, folic acid levels, and the C677T MTHFR gene polymorphism [10–12]. However, plasma homocysteine levels in BRVO patients were significantly positively correlated with macular retinal thickness at various time points after BRVO [13]. Therefore, the current study cannot prove that high plasma homocysteine level is an independent risk factor for BRVO [14]. The changes in plasma homocysteine levels in patients with BRVO from the acute phase to the convalescent phase after venous occlusion may reflect the influence of Hcy levels [15], the likelihood of the disease itself. In the SNN network structure, the structure of Kohonen network is used to introduce the multiorder parameter mechanism, and the SOM learning mechanism based on multiwin elements is constructed to realize the multiorder parameter domination mechanism and the multiobjective oriented learning method [16]. The improved SNN consists of an input layer, an order parameter layer, and an output layer [17]. The number of neurons in the input layer is equal to the feature dimension [18]. The order parameter layer based on the Kohonen network contains M*∗*M neurons, forming a square matrix [19–21].

In target recognition, sometimes, there are multiple identical or similar copies of the target to be recognized in the image, and it is difficult to classify and estimate by traditional methods. In this case, it is necessary to use the SOM network to separate multiple targets and use the multiple order parameters in the improved SNN to pair the target [22]. Orientation: recognition of a single target, isolating multiple copies of an image or identifying multiple different targets. In the feature space of the image, the SOM network uses similar features in the image, such as pixel position, color, and texture, to find similar vectors through clustering for regional division, and the pixels are distributed around the center of a class after clustering. The purpose of this study is to further study the correlation between branch retinal vein occlusion and arteriosclerosis by quantitatively measuring retinal vessel diameter and choroidal thickness, to analyze the correlation between different TCM syndrome types of nonischemic BRVO and retinal arteriosclerosis, and to provide theoretical basis for clinical nonischemic BRVO TCM syndrome types and traditional Chinese medicine treatment, so as to reflect its clinical application value. In order to solve the single fixed structure of traditional SNN and poor scalability, combined with the Kohonen layer structure in the self-organizing mapping network, an improved collaborative neural network model is proposed.

## 2. Quantitative Diagnosis of TCM Syndrome Classification of Arteriosclerosis

### 2.1. Diagnostic Criteria

RVO is divided into ischemic and nonischemic:

Ischemic RVO has severe visual loss, relative pupillary block, a large number of nonperfused areas in FFA, optic disc, and retinal neovascularization, and retinal veins are highly tortuously dilated, extensive hemorrhage, and multiple cotton wool spots under ophthalmoscope; nonischemic RVO has milder visual loss, no relative pupillary block, less bleeding, no cotton wool spots, few or no capillary nonperfusion areas in FFA, and no retinal neovascularization in the optic disc.

  Grade 1: mild thinning of arterioles, widening of reflective bands, mild or no arteriovenous crossing changes;
  Grade 2: more obvious narrowing of arterioles and widening of reflective bands, more obvious arteriovenous indentation;
  Grade 3: arterioles are copper-like, with obvious changes in arterial and venous compression;
  Grade 4: arterioles are silver filaments, severe arteriovenous cross compression changes.

In this study, referring to the “Traditional Chinese Medicine Diseases Diagnosis and Treatment Standards” issued by the State Administration of Traditional Chinese Medicine, 35 BRVO patients and 35 control groups were divided into three TCM syndrome types, namely, qi stagnation and blood stasis syndrome, Yin deficiency and yang hyperactivity syndrome, and phlegm and blood stasis syndrome. Syndrome of Yin deficiency and Yang hyperactivity is accompanied by dizziness, tinnitus, light head and feet, hot flushes, insomnia, irritability, soreness and weakness of waist and knees, red tongue with little coating, and thin pulse. Phlegm and blood stasis syndrome has a longer course of disease, obvious fundus edema and exudation, or cystoid macular edema. Among the 35 patients with BRVO, the most common syndrome type was qi stagnation and blood stasis type, 22 cases, accounting for 63% of the total; 11 cases of yin deficiency and yang hyperactivity type, accounting for 31 of the total; 2 cases of phlegm stasis type, accounting for 6% of the total. The TCM syndrome types of BRVO patients are as follows: Qi stagnation and blood stasis syndrome > Yin deficiency and Yang hyperactivity syndrome > Phlegm and blood stasis syndrome. Peng Qinghua believes that this disease is a typical blood stasis syndrome in ophthalmology. After the branch or central vein is blocked, the blood in the vessel does not run smoothly and overflows outside the vein, causing fundus hemorrhage, as shown in Figure 1.

It shows that there is no significant difference in retinal arteriovenous diameter and retinal arteriosclerosis in BRVO patients regardless of qi stagnation and blood stasis syndrome, yin deficiency and yang hyperactivity syndrome, and phlegm and blood stasis syndrome. Therefore, this study is a retrospective study, only limited TCM symptoms and signs can be obtained from the patient's hospitalization data, and a more detailed TCM syndrome element scale cannot be formulated. In the process of TCM syndrome classification, it can only be roughly classified, so it needs to be improved in future research.

In this study, the BRVO group was compared with the control group, and the BRVO group was compared with the healthy eye, and the pairwise comparison results of CRAE and AVR were statistically significant (*P* < 0.05), indicating that the retinal arteries of the BRVO patients' eyes were significantly different. The diameter of the tube decreases, and the ratio of arteriovenous decreases; that is, the retinal arteries become thinner, and the degree of retinal arteriosclerosis increases; and in the BRVO group, the ratio of retinal arteriovenous ratio is less than 2/3 of the total number of patients, accounting for 62.9%, and the healthy eyes in the BRVO group and in the normal control group, the ratio of retinal arteriovenous ratio less than 2/3 accounted for 5.7% of the total population, and the proportion of retinal arteriosclerosis in eyes with BRVO was significantly higher than that in the contralateral healthy eyes and the normal group. It indicated that gender, age, subfoveal retinal thickness, and choroidal thickness in this study could not be used as factors affecting the occurrence of retinal arteriosclerosis in eyes with BRVO. This article is the first preliminary study on the related factors of arteriosclerosis in eyes with BRVO, and it is necessary to use different statistical methods to conduct research on larger samples and more related factors.

In order to further study the related factors of retinal arteriosclerosis in BRVO eyes, age, gender, SFCT, CFT, and retinal arteriosclerosis in the BRVO group were analyzed. In this study, there were a total of 35 patients with 35 eyes in the BRVO group: the oldest patient was 81 years old, the youngest patient was 37 years old, and the average age was (60.74 ± 9.63) years old; there were 17 males with 17 eyes, 18 females with 18 eyes, male and female. The ratio was 1 : 1.1; the mean SFCT value of the affected eye was (259.46 ± 92.74) *μ*m; the mean CFT value of the affected eye was (488.51 ± 169.87) *μ*m. The correlation between retinal arteriosclerosis and age, gender, SFCT, and CFT in these 35 eyes with BRVO was analyzed, and binary logistic regression was used to draw the conclusion: whether retinal arteriosclerosis occurred in eyes with BRVO was related to gender, age, and SFCT, and there was no significant correlation between CFT (*P* > 0.05).

### 2.2. Hierarchical Collaborative Neural Network Based on Adaptive Resonance Theory

This chapter will be compatible with the design characteristics of the order parameter layer of the SNN in the network construction stage and use the redundant neurons of the order parameter layer to learn new class patterns. The specific method is as follows: first, the adaptive resonance theory is used as the guiding ideology, and the ART network architecture is used to compare the matching degree between the input source data and the existing prototype mode, and the matching degree is used as the basis for judging the new type of mode; using the network learning mechanism, the new model is guided to the redundant neurons in the order parameter layer to construct a new winning element as the representative of the new model class; and a highly robust new class learning method using the redundancy of the order parameter layer is proposed. To realize continuous learning in the network, for the problem of new class discovery, the SOM-oriented ART technology is proposed to realize the selection of ART matching degree threshold, so that the network can enhance the network's ability to classify new class data by itself through continuous learning. In addition to the fundus manifestations of Qi stagnation and blood stasis syndrome, patients with qi stagnation and blood stasis syndrome also have eye distention, headache, chest and flank pain, or emotional depression, lack of appetite, belching, tongue and pulse characterized by red tongue with ecchymosis, thin white fur, and stringy or astringent pulse.

It does not need to learn to classify objects in advance, and the encoding of environmental information is spontaneously generated in the neural network. It is a neural network that can self-organize and encode stable patterns that can respond to arbitrary sequence input patterns in real time. Modify the matching pattern when the new input vector is similar to the existing pattern, and create a new pattern when the new input vector is not similar to the existing pattern. ART theory is divided into three categories: ART1, ART2, and ART3. Among them, ART1 deals with discrete information, while ART2 deals with binary and analog information. ART3 can perform hierarchical search. SNN's new class discovery technology plans to use the ART1 model and apply and further process it, so as to complete the discovery of new class prototype models, as shown in Figure 2.

The order parameter layer of SNN maintains excessive order parameter neurons in the network construction stage, so after the network completes the current learning task, there will still be a considerable number of neurons in the order parameter layer that are always inactive. These neurons are called redundant order parameter neurons. A redundant order parameter neuron is defined as follows: for an order parameter neuron *ξr*, if the corresponding prototype pattern **vr** of the neuron is multiplied by the input sample at any time, its value is lower than the threshold *θ*, that is, **vqn**(**t**) < *θ*, and we call this neuron a redundant order parameter neuron. When all neurons in the network have been occupied, and new classes still need to be added to the network order parameter layer, the following methods are used to add neurons to the network, as shown in Figure 3. According to the arrangement between *d* and *e*, there are two ways to add redundant nodes, and the redundant nodes added become a relative row or column of neurons in the network. After adding redundant nodes, the weights on the neurons between the *d* and *e* nodes are initialized to the mean of the weights on the *d* and *e* neurons.

1. The first step, according to the ART process, when the network needs to add nodes, calculate the error node *e* in the network topology. The calculation method of *e* is *e*=argmax(∑‖*xi* − *wi*‖*xi* ∈ *Xc*), where *Xc* is the input vector mapped to the *i*-th in the network A subset of nodes, *wii*-th. The weights on each network neuron and all the corresponding forward weights are connected, and the neuron with the largest distance between the weight and the input vector is calculated.
2. In the second step, after selecting the error node *e*, calculate the distance between the weight on the error neuron node *e* and the weight on the adjacent neuron, select the most dissimilar neuron in the neighborhood of *e* Meta node, and determine the node with the largest distance as *d*, and the calculation method is *d*=argmax(‖*we* − *wi*‖), where *wi* is the weight on the neurons in the neighborhood of *e*.
3. The weights of are initialized to the new pattern vector learned by the ART process. After adding redundant nodes, in order to prevent the network from not converging, the network resets the learning rate and network neighborhood parameters to the initial values again and trains the SOM mode to achieve convergence.

### 2.3. Quantitative Diagnosis of TCM Syndrome Types

The occurrence of branch retinal vein occlusion is mostly related to dyslipidemia and retinal arteriosclerosis. Relevant studies have found that risk factors for retinal vein occlusion include hypertension, arteriosclerosis, and increased blood viscosity. Retinal arteriosclerosis is the most important risk factor for branch vein occlusion, accounting for the first cause of branch vein occlusion, up to 86.4%, followed by hypertension, accounting for 68.0%. The central retinal artery is different from the large arteries in other parts of the human tissue. Its inner elastic layer is only a single layer, and the muscle layer is also a single layer of muscle fibers. After the second branch, the inner elastic layer disappears, and the muscle layer is no longer continuous. Therefore, all retinal arteries are small arteries. The pathological characteristics of arteriosclerosis are degenerative, noninflammatory, and proliferative changes in arteries, resulting in hardening of the wall and loss of elasticity and narrowing of the lumen. Retinal arteriosclerosis is mainly caused by the proliferation of retinal arterial medial muscle cells, the later cell degeneration, and the formation of hyaline degeneration of muscle fibers. In the case of arteriosclerosis, adjacent or intersecting arteries compress veins with weaker walls, narrowing the lumen of the vein, edema, and hyperplasia of endothelial cells under pressure, further narrowing of the lumen and obstruction.

Retinal arteries and veins, due to anatomical reasons, the central retinal arteries and veins are close to each other at the cribriform plate, and there is a common sheath at the intersection of retinal arteries and veins. The general retinal artery-to-vein ratio is 2/3. When arteriosclerosis occurs, the arterial diameter becomes thinner, and the arteriovenous ratio decreases to less than 2/3. By evaluating the correlation between retinal microvascular diameter (including CRAE, CRVE, AVR) and macrovascular arteriosclerosis, the macrovascular arteriosclerosis was evaluated by pulse wave velocity (PWV) and aortic reflection wave enhancement index (AIx) and obtained. Compared with normotensives, hypertensive patients had significantly increased PWV and AIX and decreased CRAE and AVR.

## 3. Results and Analysis

### 3.1. Experimental Dataset

The experimental data set used in this paper adopts Extended MNIST (EMNIST), because MNIST is well known, but the accuracy of the classifier on MNIST is already very high, and a good data set should be more challenging, so EMNIST is used here.

On the dataset interface, the processing method of this dataset is consistent with that of MNIST. Here, we will focus on the classification method of EMNIST. Because of language and usage habits, there are also differences in case between letters, because some letters are basically difficult to distinguish between uppercase and lowercase handwriting. All these letters are merged here to form a new category. There are 15 classes [C, I, J, K, L, M, O, P, S, U, V, W, X, Y, Z], so 47 classes are left in the end.

EMNIST is mainly divided into the following 5 subdatasets:

  By Class: a total of 814,255 images, 62 classes; reclassify the number of images in the training set and test machine compared to NIST.
  By Merge: a total of 814255 images, 47 categories, compared with NIST; the number of images in the training set and the test machine are reclassified.
  Balanced: a total of 131,600 images, 47 categories; each category contains the same amount of data, 2,400 for training set and 400 for test set for each category.
  Digits: 28,000 images in total, 10 categories; each category contains the same amount of data, 24,000 for training set and 4,000 for test set.
  Letters: 145,600 sheets in total, 26 categories; each category contains the same data, 5,600 sheets for training set and 800 sheets for test set for each category.
  MNIST: a total of 70,000 images, 10 categories; each category contains the same amount of data.

The pictures in the data set are 28*∗*28 dimensions. Since the position of the handwritten characters in the picture is not fixed, first, a sliding window of size 24*∗*24 is used, and the step size is set to 1, and the features are extracted from the image, and each sample can get 25 pictures. For subgraphs of the same category, the balanced data set of EMNIST is used here to avoid possible data imbalance problems. The sample vector is a 24*∗*24-dimensional vector, of which there are 2,820,000 images in the training dataset and 470,000 images in the test dataset. During training, batch training is adopted, and the batch size of each batch is 10,000; that is, 10,000 samples are randomly selected from the training set for training. The network convergence situation is shown in Figure 4. It can be seen from the table that the SNN model based on ART and SOM has a higher recognition accuracy than the baseline linear classifier and the classic SVM classifier. There is a certain improvement. Compared with the improved SNN method of SOM + SNN in Chapter 3, the average recognition rate is increased by 13.09%.

Use the test set shown in Figure 5. This is because the hierarchical structure is adopted in the network structure, and the network can be generated without increasing the complexity. More neuron nodes make the subclasses corresponding to the classification more refined, and the network recognition effect is better. In addition, the local optimal search is used in the network model, which greatly reduces the time complexity and shortens the training time. Compared with the handwritten digit dataset MNIST, the EMNIST handwritten character dataset has a larger number of categories, and the difference between each category is small, especially with a large number of easy-to-use handwritten characters, confused samples of different classes.

Such a sample can get 64 subsamples with the same label, and the convolutional features are used as the input of our proposed improved hierarchical SNN for training. The hidden layer structure of the obtained network is shown in Figure 6. The darker and denser parts of the grid represent deeper layers and more complex subsequence parameter layers in the network. Generally speaking, the more subclasses of the same classification represented by each leaf neuron node in the order parameter layer network in the network, the more complex the network level, and the more refined the effective features learned by the network. In the experiments, the first three layers of the pretrained CNN are used to extract convolutional features.

The time complexity of the method in this paper is shown in Figure 7. The table shows the time complexity of each layer in the network, where N is the number of training samples, *m* is the sample dimension, W is the number of weights, and C is the number of classifications. This is consistent with the majority of the patients with Qi stagnation and blood stasis syndrome in this study. There was no significant difference in the comparison of CRAE, CRVE, and AVR of three different TCM syndrome types in BRVO group (*P* > 0.05).

In order to compare the time complexity and space complexity of the method in this paper and other deep learning methods, as shown in Figure 8, the table shows the comparison of the parameter scale and calculation amount of the method in this paper and different classifiers. The amount of computation corresponds to the time complexity of the network, which is the length of network training and running time, and the number of parameters corresponds to the space complexity of the network, which is the amount of GPU memory occupied by the network. In the convolutional neural network, because there are a large number of fully connected layers in the model design, when the dimension of the convolutional feature obtained by the network after multiple convolutions is large, the scale of the parameters in the network is often very large, which is also a lot of related research, the reason why the convolutional neural network needs to design multiple convolutional layers to convolve the input data. In the method of this paper, a convolutional layer is used to extract convolutional features in the feature extraction stage of the network input data, and then the hierarchical network structure is used to avoid the computational difficulty caused by the large scale of the hidden layer of the SNN network and reduce the size of the network. The time complexity of the network improves the network performance.

## 4. Quantitative Analysis of TCM Syndrome Types

After extracting convolutional features, in order to verify the performance gap between the method proposed in this chapter and other methods, the SNN network and other convolutional neural networks are used for classification and recognition. The other three classifier models are AlexNet and VGG-16 Net. The specific results are shown in Figure 9.

Compared with the CNN method, the effect of classifying convolutional features by extracting convolutional features and then using SNN is improved to a certain extent. In the pattern recognition problem in the case of multiclassification and complex samples, through reasonable structure and parameter optimization, the method in this paper can also meet the practical requirements. The blood supply of the choroid mainly comes from the short posterior ciliary artery, which has many blood vessels and a large blood volume, accounting for about 64%–84% of the blood flow of the eye. The choroid is mainly composed of blood vessels, and its thickness varies greatly with the degree of vascular filling. The choroidal blood circulation mainly supplies the nutrition of the outer layer of the retina and the anterior optic nerve of the cribriform plate and is the only source of nutrition for the fovea of the macula, which plays an important role in maintaining the physiological function of the retina. Choroidal thickness is also affected when structural and functional lesions of the eye occur. The thickness of the choroid is closely related to age, blood supply, and diopter. In addition, local diseases of the eye and systemic factors can also reduce the blood flow of the choroid, resulting in a decrease in the thickness of the choroid. Choroidal blood flow velocity is negatively correlated with age. The older the age, the lower the choroidal blood flow velocity. In addition, the density and diameter of blood vessels also gradually decrease. In a study on the macular choroidal thickness of Chinese people, the macular choroidal thickness and its influencing factors were analyzed in 360 eyes of 180 volunteers, and the CT value of the Chinese macular region was (262.78 ± 84.38) pm, as shown in Figure 10. The thickness of the side healthy eye increased. There was a statistically significant difference in SFCT between the eyes with BRVO and the control group (*P* < 0.05); that is, the choroid was thickened in the eyes with BRVO compared with the normal eyes, indicating that the thickness of the choroid in the eyes with BRVO was higher than that of the normal eyes.

Diopter was the main influencing factor of macular CT in <60 years old, and age was the main influencing factor of macular CT in ≥60 years old. Choroidal thickness is closely related to age and diopter. There are many studies on the relationship between wet macular degeneration (wAMD), central serous chorioretinopathy (CSC), idiopathic polypoid chorioretinopathy (PCV), high myopia, glaucoma, and other eye diseases and choroidal thickness in the literature. Few studies have investigated the relationship between branch retinal vein occlusion and choroidal thickness. In this study, there was a statistically significant difference in SFCT between the BRVO group and the healthy eyes (*P* < 0.05); that is, the choroid was thickened in the BRVO eyes compared with the healthy eyes, indicating that the choroid thickness of the BRVO eyes was higher than that of the other eyes. According to the literature, a variety of eye diseases can cause changes in choroidal thickness: central serous chorioretinopathy causes increased choroidal thickness, which is based on the loss of continuity of the retinal pigment epithelium, and the choroid is hyperperfused. Destruction occurs because of each other; the choroidal thickness of patients with idiopathic macular hole is significantly thinner than that of the normal group, and the influence of choroidal thickness is mainly due to the decrease of choroidal blood flow velocity and blood flow; Vogt-Koyanagi Harada syndrome is self-induced due to immune response, genetically related panuveitis, immune response caused by inflammatory mediators, and autoantigens thickening the choroid.

## 5. Conclusion

The main branches of the human ophthalmic artery are the central retinal artery, the posterior ciliary artery, and the branches of the ophthalmic muscle, and the human ophthalmic artery is the branch of the internal carotid artery. Atherosclerotic plaques cause vascular stenosis, insufficient cerebral blood supply, local thrombosis, or the rupture of plaques and fragments fall off, resulting in insufficient blood supply to the eye or embolism and other bleeding disorders. Elevated blood lipids, increased blood viscosity, slowed hemodynamics, local retinal circulation disorders, and increased capillary permeability are also the causes of BRVO. It is of great significance to further study the correlation between branch retinal vein occlusion and arteriosclerosis, to analyze the correlation between different TCM syndrome types of nonischemic BRVO and retinal arteriosclerosis, and to provide theoretical basis for clinical nonischemic BRVO TCM syndrome types and traditional Chinese medicine treatment, so as to reflect its clinical application value. In order to solve the single fixed structure of traditional SNN and poor scalability, combined with the Kohonen layer structure in the self-organizing mapping network, an improved collaborative neural network model is proposed. This paper studies the network training method and operation convergence and analyzes the converged network and the pattern classification results obtained by the network. The results of our proposed improved model on the MNIST dataset can achieve the same level of current state-of-the-art machine learning classifiers in recognition accuracy with a smaller network size and network complexity.

In the future, a convolutional layer is used to extract convolutional features in the feature extraction stage of the network input data, and then the hierarchical network structure is used to avoid the computational difficulty caused by the large scale of the hidden layer of the SNN network.

## Figures and Tables

**Figure 1:** Correlation regression analysis of arteriosclerosis in eyes with BRVO.

**Figure 2:** SNN network design for ART matching degree calculation method.

**Figure 3:** Schematic diagram of adding redundant nodes to the network order parameter layer.

**Figure 4:** Schematic diagram of network training convergence.

**Figure 5:** Comparison of EMNIST experimental results.

**Figure 6:** Visualization of the order parameter layer structure.

**Figure 7:** Time complexity of our method.

**Figure 8:** Comparison of parameter scale and computational cost between our method and different classifiers.

**Figure 9:** Comparison of recognition rates between SNN and different classifiers supported by CNN.

**Figure 10:** Comparison of CFT between healthy and affected eyes in BRVO group.

## Data Availability

The data used to support the findings of this study are available from the corresponding author upon request.
